# Real-World Evidence of Traditional Chinese Medicine (TCM) Treatment on Cancer: A Literature-Based Review

**DOI:** 10.1155/2022/7770380

**Published:** 2022-06-29

**Authors:** Linjia Peng, Ke Zhang, Yujie Li, Lianyu Chen, Huifeng Gao, Hao Chen

**Affiliations:** Department of Integrative Oncology, Fudan University Shanghai Cancer Center, Shanghai, China

## Abstract

While randomized controlled trials (RCTs) are the gold standard for evidence-based medicine, they do not always reflect the real condition of patients in the real-world setting, which limits their generalizability and external validity. Real-world evidence (RWE), generated during routine clinical practice, is increasingly important in determining external effectiveness of the tightly controlled conditions of RCTs and is well recognized as a valuable complement to RCTs by regulatory bodies currently. Since it could provide new ideas and methods for clinical efficacy and safety evaluation of traditional Chinese medicine (TCM) and high-quality evidence support, real-world study (RWS) has received great attention in the field of medicine, especially in the field of TCM. RWS has shown desirable adaptability in the clinical diagnosis and treatment practice of traditional Chinese medicine. Consequently, it is increasingly essential for physicians and researchers to understand how RWE can be used alongside clinical trial data on TCM. Here, we discuss what real-world study is and outline the benefits and limitations of real-world study. Furthermore, using examples from TCM treatment on cancer, including Chinese herbal medicine, acupuncture, moxibustion, integrated TCM and Western medicine treatment, and other treatments, we elaborate how RWE can be used to help inform treatment decisions when doctoring patients with cancer in the clinic.

## 1. Real-World Study (RWS)

### 1.1. What Is Real-World Study (RWS) and Real-World Evidence (RWE)?

Real-world study refers to the process of the collection of data (real-world data) related to the health of research subjects in a real-world setting or aggregated data derived from preset clinical questions and through analysis, to obtain medication utilization, potential benefits, and benefit-risk clinical evidence. Real-world data refer to diverse data collected on a routine basis related to physical conditions of patients besides diagnosis, treatment, and care. Not all real-world data can become real-world evidence after analysis, and only real-world data that satisfy applicability can generate real-world evidence. Real-world evidence refers to clinical evidence on the use and potential benefit-risk of a drug obtained through appropriate and adequate analysis of applicable real-world data, including evidence from retrospective or prospective observational studies or interventional studies such as pragmatic randomized controlled studies [1]. RWS is characterized by the use of large-scale sample data, relaxation of inclusion and exclusion criteria, long-term follow-up, attention to the real clinical setting, and selection of different interventions according to the patient's actual condition and willingness, as well as the selection of broadly clinically significant indicators to evaluate outcomes [2, 3]. RWS has been widely used in the research of long-term outcome evaluation of postmarketing drugs, patient compliance, disease characteristics, rare subtypes of cancer, and special populations [4–8].

### 1.2. Benefits and Limitations of Real-World Study

For a long time, it has been firmly convinced that RCT is the most effective research mean to verify causality and the gold standard for testing treatment effects which drive the high internal authenticity and accuracy conclusions of research studies [4, 9, 10]. However, with the poor extrapolation of RCT and the sample size limited by different diseases, RCT requires a lot of financial, materials, labor, and time cost investment which cause both operability and economic benefits difficult to attain [9, 10]. Cohort studies and case-control studies are also widely used in TCM clinical research, but they also have different benefits and limitations. Case-control studies are easy to organize and carry out and can simultaneously study the association between multiple factors and a disease. They are especially suitable for exploratory etiological studies and do no harm to the study subjects. On the other hand, it is difficult to avoid selectivity and recall bias when selecting subjects and obtaining previous information. The authenticity of information is difficult to guarantee, the sequence of exposures is often difficult to determine, and the confounding effects are difficult to control. When it comes to cohort studies, the benefits are as follows: first, subjects were grouped according to their exposure and followed up before the occurrence of disease, and the data obtained were complete and reliable without recall bias. Second, the time sequence of exposure factors and diseases is clear, so the ability to demonstrate the causal relationship is strong. Third, it can directly estimate the strength of the association between exposure and disease as well as help understand the natural history of disease. Moreover, the limitations are as follows: first, the organization and implementation are difficult, time-consuming, laborious, and costly. Second, it is not suitable to study diseases with a very low incidence. Third, because of the long follow-up time, it is prone to loss of follow-up bias. Fourth, it requires high design requirements and complicated data collection and analysis.

Traditional clinical trials play a very vital role in promoting the modernization and standardization of traditional Chinese medicine, but traditional Chinese medicine emphasizes the integration of heaven and earth, respects individual differences, and follows the characteristics of syndrome differentiation for treatment, which determines that the types of studies mentioned above are difficult to reflect the curative effect and characteristic advantages. Based on real-world settings, which generalizes the conclusions, the emergence of RWS compensates for the insufficiency of RCT [7]. Therefore, in the evaluation of TCM efficacy, both scientific rigor and flexibility should be given to reflect the objective reality. RWS can fully reflect these characteristics, providing a new path and mean for TCM efficacy evaluation and evidence accumulation. In addition, RWS can also be used for paradigm and program optimization of complementary advantages of integrated traditional Chinese and Western medicine to establish evidence for clinical efficacy improvement. Finally, it can provide the basis for early clinical research to develop new treatment methods. Although RWS has many advantages, this open, nonrandom research method also has some limitations: First, because of the lack of randomization and low internal authenticity, the reliability of the results will be questioned. Second, observer bias affects the quality of the research results, especially the differentiation of TCM syndrome and personal experience, autonomy, and randomness. Third, patients' compliance may not be high due to long follow-up time. Fourth, there are many confounding factors, so it is not only difficult to distinguish the effectiveness of a single component in the overall intervention but also the results of the study may be close to meaningless. Fifth, to a certain extent, because it is an observational study and no intervention measures are taken, its research effectiveness has a certain lag [11]. In addition, it requires a large number of research samples and even multicenter events and has high difficulty in data collection, huge workload, strong data heterogeneity, and higher requirements on statistical methods than traditional research, and most of them are retrospective analysis or post hoc analysis, so how to ensure the effectiveness of research evidence is a challenge. Nevertheless, RWS can complement other types of research to further supplementing evidence of efficacy [1, 4, 12].

Table 1 summarizes the distinction between real-world studies and randomized controlled trials, cohort studies, and case reports.

## 2. Real-World Evidence from Traditional Chinese Medicine on Cancer

Clinical efficacy and safety have always been the core content of research in the field of traditional Chinese medicine. However, with the continuous deepening of research as well as its limitations, RCTs have been unable to meet the clinical demand of traditional Chinese medicine which is considered with unique diagnostic advantages. In recent years, how to scientifically and objectively evaluate the validity of traditional Chinese medicine in a real-world setting has become a hot topic in clinical research. As an important supplement to randomized controlled trials, real-world study is one of the approaches in line with the scientific research paradigm of TCM clinical research. Based on the characteristics of clinical diagnosis and treatment of traditional Chinese medicine, it collects a large amount of real-world data, as well as incorporates clinically meaningful outcomes, so as to mine and evaluate the efficacy and safety of traditional Chinese medicine in the real world.

Traditional Chinese medicine has remarkable effects on cancers in the clinical practice, either directly inhibiting the occurrence and development of tumors, or reducing the side effects caused by chemotherapy and radiotherapy, or reducing the dosage of other therapies. Kuo conducted a real-world analysis of 582,799 adult cancer patients in Taiwan based on whether they used traditional Chinese medicine. The main analysis was the use of traditional Chinese medicine, as well as specific medical visits. After the adjustment of age, gender, urbanization of residence, occupation, annual medical center visit, and annual nonmedical center visit, adjusted hazard ratios (aHR) for mortality were significantly lower among TCM users than those who do not get TCM. This study indicates that more attention should be paid to the use of traditional Chinese medicine in the clinical diagnosis and treatment of cancer patients [13].

Since acupuncture, moxibustion, and other treatments of TCM are rarely used in the treatment of tumors alone, they are mainly used to treat the adverse reactions and tumor-related complications. Therefore, this paper mainly focuses on the discussion of Chinese herbal medicine.  Table 2 summarizes the contents related to the treatment of tumors by acupuncture and other therapies. In addition, the integrated TCM and Western medicine treatment in the real-world clinical practice is summarized in Table 3. Next, we will conduct literature mining for common clinical tumors and sort out the antitumor effects of Chinese herbal medicine under real-world conditions. The results are summarized in Table 4. Moreover, Table 5 demonstrates the types of syndrome differentiation of common tumors.

### 2.1. Respiratory System Cancer

Lung cancer is the most common malignant tumor of the respiratory system, accounting for most of the tumors of the respiratory tract [14]. Buzhong Yiqi Decoction, Xiangsha Liujunzi Decoction, Baihe Gujing Decoction, Bei-Mu (BM), Xing-Ren (XR), and Ge-Gen (GG) are the most commonly used Chinese herbal formulas and Chinese medicines for the treatment of lung cancer, respectively [15]. A real-world study led by Li included 1988 patients with newly diagnosed locally advanced metastatic lung adenocarcinoma between 2006 and 2012 who received first-line therapy gefitinib or erlotinib as well as the Chinese herbal medicine as an adjuvant treatment. Compared with patients who did not receive Chinese herbal medicine, the mortality rate of patients who used Chinese herbal medicine for ≥180 days was significantly reduced, which means that in patients with advanced lung adenocarcinoma treated with first-line TKIs, adjuvant Chinese herbal medicine treatment could improve the overall survival rate and progression-free survival rate [16]. Additionally, another study showed that Qingzao Jiufei Decoction was an effective decoction in reducing lung cancer mortality in a real-world setting [17].

### 2.2. Digestive System Cancer

The most common tumors of the digestive system are colorectal cancer, pancreatic cancer, liver cancer, intrahepatic bile duct cancer, and gastric cancer [14]. A total of 13,943 pancreatic cancer patients were divided into two groups according to whether they took Chinese herbal medicine (mainly Chinese medicine Hedyotis diffusa and Chinese herbal formula Xiangsha Liujunzi Decoction) in a real-world setting. The results showed that pancreatic cancer patients who had used complementary Chinese herbal medicine had a better prognosis and those who received CHM for more than 90 days had a significantly lower hazard ratio for mortality than non-CHM users [18]. In addition, a real-world study of traditional Chinese medicine in the treatment of liver cancer analyzed the commonly used Chinese herbal medicine treatments in liver cancer patients and their impact on the survival of liver cancer patients. It turns out that Jiawei Xiaoyao San and Chaihu Shugan Decoction were the most effective Chinese herbal formula to improve the overall survival, as well as significantly improve the survival rate of patients with liver cancer [19]. By observing the clinical efficacy and adverse reactions of patients with advanced colorectal cancer treated with Jianpi Jiedu Tongluo formula combined with tegafur maintenance under real-world conditions, the results indicated that this scheme can improve the quality of life of patients and prolong the disease-free survival of the disease [20]. Regarding the study of gastric cancer, the results of the study proved that complementary traditional Chinese medicine (mainly Chinese herbal medicine Herba Hedyotidis Diffusae and Xiangsha Liujunzi Decoction) can significantly improve the survival rate of gastric cancer patients [21]. As for metastatic gastric cancer, a study on the effect of traditional Chinese medicine, especially Fuzheng Jiedu therapy, on the overall survival rate and progression-free survival rate of patients was conducted in a real-world setting, thus exhibiting that the most commonly utilized medicine in this therapy are Chinese herbal formula Shenmai and compound Kushen injections which can significantly improve the survival rate of patients with metastatic gastric cancer [22].

### 2.3. Breast Cancer

Breast cancer (BC) is the second most commonly diagnosed cancer in women in the United States and a prime reason for death in women globally [14]. A real-world study from Taiwan included 79,335 breast cancer patients who were divided into two groups based on whether they took more than 80 grams of Danshen within 28 days after diagnosis. The findings suggest that higher doses or longer use of Danshen has a protective effect in breast cancer patients [23]. Besides, according to whether they used traditional Chinese medicine while receiving hormone therapy, estrogen receptor (+) breast cancer patients were divided into two groups. The use of TCM did support the potential advantage of TCM in breast cancer-related mortality, while did not show significant impact on adherence to HT [24]. Tamoxifen is a common drug for patients with estrogen receptor-positive breast cancer [25–27], but it is easy to induce endometrial cancer and various adverse reactions [26]. Jia-Wei-Xiao-Yao-San and Shu-Jing-Huo-Xue-Tang significantly improved the overall survival rate of estrogen receptor-positive breast cancer patients and reduced the risk of tamoxifen-induced endometrial cancer [28].

### 2.4. Other Cancers

Chinese herbal medicine also plays a significant role in treating other cancers. As for cervical cancer, Bai-Hua-She-She-Cao (Herba Oldenlandiae, synonym: Herba Hedyotis diffusae) and Jia-Wei-Xiao-Yao-San were the most commonly used single-flavor Chinese medicine and Chinese herbal formula, respectively. After treatment, compared with cervical cancer patients who did not use Chinese herbal medicine, the survival rate of cervical cancer patients who took Chinese herbal medicine was significantly improved [29]. One study performed a real-world retrospective cohort study of head and neck cancer (HNC) patients between 2001 and 2011 using the Taiwan National Health Insurance Research Database. The Cox regression model was used to determine the correlation between Chinese herbal medicine use and survival outcomes. The results demonstrated that the application of Chinese herbal medicine was significantly associated with a 32% reduction in all-cause mortality. Patients who took Chinese herbal medicine for a long time had lower mortality [30]. By taking whether or not to take Chinese herbal medicine as an exposure factor, Xu collected 595 patients with stage III-IV esophageal cancer and divided them into two groups based on taking or not taking Chinese herbal medicine. Analyzing the follow-up survival time and prognostic factors of the patients, the results showed that Chinese herbal medicine could prolong the survival time of patients with stage IV esophageal cancer and taking Chinese herbal medicine was an independent factor for the survival time of patients with stage IV esophageal cancer [31].

## 3. Discussion

In China, more than 4 million people are diagnosed with cancer every year, and with its morbidity and mortality, it ranks first in the world and has become a major public health problem that seriously endangers human health [32]. Conventional treatment options include surgical resection [33], chemotherapy [33], and radiotherapy [34], and new treatment options including immunotherapy [34–37] and targeted therapy [38–42] are continuously generating and developing. Despite present diverse desirable effects, they also bring different degrees of recurrence and side effects. As the birthplace and most widely used country of traditional Chinese medicine, in fact, more than 80% of cancer patients in China have received traditional Chinese medicine treatment more or less, indicating that traditional Chinese medicine has an irreplaceable position and importance in the treatment of malignant tumors. Traditional Chinese medicine has abundant experience in the treatment of cancers and has definite curative effect on a variety of common tumors in the clinic. In addition, traditional Chinese medicine also exhibit a certain alleviation effect on the side effects caused by surgery, chemotherapy, and other treatments and some precancerous lesions [43, 44]. A large number of studies have also proved that traditional Chinese medicine including Chinese herbal medicine, acupuncture, and moxibustion as well as other treatments exert their antitumor effects from multiple perspectives and multiple targets [44–52]. The antitumor mechanism of Chinese herbal medicine is shown in Figure 1.

Real-world study has received global attention since its inception due to its consistency to clinical practice [53]. China, the United States, and European countries have successively passed a series of policy bills to support the development of RWS [53–56]. Undoubtedly, the concept of the real world is extensively accepted by clinical researchers and RWS has set off a global research boom [57]. RWS is closely linked with human life and health in the field of medicine which is clinical problem-oriented research that involved all stages of the diagnosis and treatment process such as disease etiology, diagnosis, treatment, prognosis, and clinical prediction models, which will overwhelmingly improve the quality of life and health of patients.

Despite there are already reviews on the clinical efficacy and mechanism of TCM in the treatment of cancer, the clinical efficacy of TCM in the real world remains to be studied [58]. In the field of traditional Chinese medicine, RWS is mostly used to evaluate the effectiveness and safety of prescriptions that combine traditional Chinese and Western medicine or to analyze the relationship between “drug-drug,” “drug-syndrome,” and “disease-syndrome.” In terms of research methods, the most widely applied one is observational study. The statistical analysis method is essentially the same as that of traditional clinical research, but the needs to be focused on the control of bias and confounding factors. From the perspective of research needs, RWS is a new research method that is not a substitute for existing types of studies but a supplement [1, 57]. However, it is expected to look for more evidence and clues to solve clinical problems in the real-world setting outside the nonrigorous RCT conditions. Because the diagnosis, treatment, and prognosis of different tumors are quite different, real-world research has a wonderful match with traditional Chinese medicine on clinical research and treatment on tumors. On the one hand, it can restore the clinical efficacy of traditional Chinese medicine in the treatment of tumors, and on the other hand, it can reduce the medical burden of patients to varying degrees.

All in all, the application of RWS in the field of traditional Chinese medicine has great potential in the future and will dispose of more problems closely related to clinical practice. We expect that better design and analysis methods can be discovered, adjusted, and applied, and the limitations and problems of the application of RWS can be better solved.

## Figures and Tables

**Figure 1:** The antitumor mechanism of traditional Chinese medicine.

**Table 1:** The distinction between real-world study and randomized controlled trials, cohort studies, and case reports.

Characteristic	Randomized controlled trials (RCT)	Real-world study (RCT)	Cohort study	Case-control study
Purpose	Focused on efficacy	Diverse research purposes, including efficacy studies	Test etiological hypotheses, evaluate preventive effects, and study the natural history of disease	Explore the cause of disease

Study population	Ideal world crowd and strict standards of inclusion and exclusion	Real-world population and broader inclusion and exclusion criteria	Exposure to study factors and control groups	People with and without the disease

Sample size	Calculated according to statistical formula, the sample size is limited	Calculated based on the real world or statistical formula, the sample size can be large or small	Calculated according to statistical formula, the sample size is required to be large	Calculated based on the study design or statistical formula, the sample size is small

Research time	Shorter (mostly end with the assessment of outcome)	Short term or long term (to obtain all treatments and long-term clinical outcomes as endpoints)	Longer research time, long follow-up time	Shorter (depends on the purpose)

Outcome	Internal validity	High external validity	Internal authenticity is not as good as RCT, and external authenticity is not as good as RWS	Both internal and external authenticity are deficient

Design	Randomization, control, prospective study	Random or nonrandom sampling, prospective or retrospective study	Prospective or retrospective or ambispective cohort study	Control, contrast

Implementation scenario	Highly standardized environment	Medical institutions, communities, homes, etc.	Medical institutions and communities	Medical institutions and communities

Data	Standardization, strict specification of the collection process	Diverse sources and high heterogeneity	Different confounding factors and bias	Different confounding factors and bias, heterogeneity

**Table 2:** Acupuncture and other treatments in the treatment of tumor-related complications and adverse reactions.

Disease or symptom	Acupuncture and other treatments	Primary outcome	Therapeutic effect
Cancer-related pain (CRP) [59]	Acupoints on the back (back-shu points)	Pain level measured with numerical rating scale (NRS)	Relieve cancer-related pain at midtreatment and posttreatment

Breast cancer-related symptom [60]	Acupuncture	Improvement and relief of symptoms	Perceived improvement in muscle pain, postsurgical pain, hot flushes, nausea/vomiting, low mood/depression, anxiety, lymphedema, and neuropathy

Breast cancer-related flushes and night sweats [61]	Auricular acupuncture	Improvement of hot flushes and night sweats (HFNS) associated with adjuvant hormonal treatments	Relief from hot flushes and night sweats

Cancer pain [62]	Acupuncture	Pain level measured with numerical rating scale (NRS) and daily opioid dose	Pain improved and opioid use decreased

Cancer-related insomnia [63]	Electroacupuncture	Insomnia Severity Index (ISI), Pittsburgh Sleep Quality Index(PSQI), sleep diary and actigraphy-derived sleep parameters, functional assessment of cancer therapy-fatigue (FACT-F), Montreal Cognitive Assessment (MoCA), and salivary levels of cortisol and melatonin	Improvements in various sleep indicators

**Table 3:** The integrated TCM and Western medicine treatment in the real-world clinical practice.

Cancer	Treatment	Primary outcome	Therapeutic effect
Hepatocellular carcinoma [64]	Jianpi Liqi Fang and transcatheter arterial chemoembolization	Karnofsky performance status and traditional Chinese medicine (TCM) syndrome scores	Serum aspartate aminotransferase levels and total bilirubin levels decreased; Fibulin-5 displayed the largest difference

Postoperative colorectal cancer [65]	Bushen-Jianpi-Jiedu decoction combined with chemotherapeutic drugs (oxaliplatin)	Progression-free survival (PFS) and Karnofsky performance score (KPS)	Prolongs the survival and improves Karnofsky performance status

Nonsmall cell lung cancer [66]	Kangliu Jiandu formula combined with chemotherapy	Improvement rate of traditional Chinese medicine syndrome, curative effect of TCM syndrome, Karnofsky performance status (KPS) score, European Organization for Research and Treatment of Cancer-Quality of Life Questionnaire-Lung Cancer	Significantly decreased the symptom area of QLQ-C30 and QLQ-LC13 score and increased the overall health status score of QLQ-C30, which were better than the control group

Breast cancer [67]	Chinese herbal medicine combined with Western medicine	Quality of life, frequency of symptom distress, and clinical safety	Higher red blood cell counts and lower liver function

Castration-resistant prostate cancer [68]	Fuyang Huayu prescription combined with chemotherapy (intravenous injection of docetaxel plus oral prednisone)	Level of serum prostate-specific antigen (PSA), Karnofsky physical condition scores, function assessment of cancer therapy-prostate (FACT-P) scores, and TCM symptom scores	Karnofsky, FACT-P, and TCM symptom scores were all markedly improved

**Table 4:** The results of TCM treatment of common tumors (types of cancer, title of literature, Chinese herbal medicine, primary outcome, and improvements in other areas).

Type of cancer	Title of literature	Chinese herbal medicine	Primary outcome	Improvements in other areas
Advanced lung adenocarcinoma	Adjunctive traditional Chinese medicine improves survival in patients with advanced lung adenocarcinoma treated with first-line epidermal growth factor receptor (EGFR) tyrosine kinase inhibitors (TKIs): a nationwide, population-based cohort study [16]	*F. thunbergii*, *O. diffusa*, and *P. grandiflorum*, Bai He Gu Jin Tang	Overall survival and progression-free survival	Increase efficacy and reduce toxicity

Lung cancer	Characteristics of Chinese herbal medicine usage and its effect on survival of lung cancer patients in Taiwan [15]	Bu Zhong Yi Qi Tang, Xiang Sha Liu Jun Zi Tang, and Bai He Gu Jin Tang; and Bei Mu, Xing Ren, and Ge Gen	The mortality hazard ratio	—

Lung cancer	Traditional Chinese medicine as adjunctive therapy improves the long-term survival of lung cancer patients [17]	Qing Zao Jiu Fei Tang, Jia Wei Xiao Yao San, Xuefu Zhuyu decoction	All-cause death	Reduction of nausea and vomiting, host immune response stimulation

Pancreatic cancer	Complementary Chinese herbal medicine therapy improves survival of patients with pancreatic cancer in Taiwan: a nationwide population-based cohort study [18]	Bai Hua She She Cao and Xiang Sha Liu Jun Zi Tang	The hazard ratio of mortality risk	Reduce gastrointestinal symptoms, anxiety, and insomnia

Liver cancer	Adjunctive traditional Chinese medicine therapy improves survival of liver cancer patients [19]	Jia Wei Xiao Yao San and Chai Hu Shu Gan Tang	All-cause mortality during the 11-year follow-up	Reduce nausea, vomiting, lipoproteinemia, chronic gastritis, and appetite loss

Middle and advanced colorectal cancer	Clinical observation on the combination of spleen detoxification and Tongluo formula with tegafur in the maintenance treatment of middle and advanced colorectal cancer in the real world [20]	Spleen detoxification and Tongluo formula	The KPS, DFS, OS, and toxic side effects	Reduce intestinal obstruction, cancer ascites, and other complications and toxic side effects of radiotherapy and chemotherapy

Gastric cancer	Complementary Chinese herbal medicine therapy improves survival of patients with gastric cancer in Taiwan: a nationwide retrospective matched-cohort study [21]	Bai Hua She She Cao and Xiang Sha Liu Jun Zi Tang	The HR of mortality risk and survival probability	Relieve cancer-related fatigue or gastrointestinal disorders

Metastatic gastric cancer	Effect of Fuzheng Qingdu therapy for metastatic gastric cancer is associated with improved survival: a multicenter propensity-matched study [22]	Shenmai and Compound Kushen injections, Shenqi Shiyi Wei Granule	Overall survival and progression-free survival	Enhance clinical efficacy and reduce adverse effects

Breast cancer	Danshen improves survival of patients with breast cancer, and dihydroisotanshinone I induces ferroptosis and apoptosis of breast cancer cells [23]	Danshen	Survival probability	Diminish the systemic cancer treatment-related adverse effects

Breast cancer	Influence of traditional Chinese medicine on medical adherence and outcome in estrogen receptor (+) breast cancer patients in Taiwan: a real-world population-based cohort study [24]	—	Evaluation of medication adherence to HT	Prevent recurrence and metastasis, delay tumor progression, and prolong survival

Breast cancer, endometrial cancer	The use of Chinese herbal medicine products and its influence on tamoxifen-induced endometrial cancer risk among female breast cancer patients: a population-based study [28]	Jia Wei Xiao Yao San and Shu Jing Huo Xue Tang	The HR for the development of endometrial cancer among CHP users	—

Cervical cancer	Adjunctive Chinese herbal medicine treatment is associated with an improved survival rate in patients with cervical cancer in Taiwan: a matched cohort study [29]	Bai Hua She She Cao and Jia Wei Xiao Yao San	Survival probability	Improve the side effects of chemo- or radiotherapy such as dysfunction of liver, diarrhea, fatigue, and pain

Head and neck cancer	The use of adjunctive traditional Chinese medicine therapy and survival outcome in patients with head and neck cancer: a nationwide population-based cohort study [30]	Gan Lou Yin	All-cause mortality during the 11-year follow-up	Attenuate toxicity and enhance the efficacy of allopathy, improving phagocytosis

Esophageal cancer	The real-world study of the clinical efficacy of traditional Chinese medicine in the treatment of III-IV stage esophageal cancer [31]	Dan Shen, Huang Qi, Fu Ling, San Qi, Wei Ling Xian, and Sheng Di	Over survival	Improve the curative effect and quality of life and reduce the adverse reaction of digestive tract and blood toxicity

**Table 5:** The types of syndrome differentiation of common tumors.

Cancer	Syndrome differentiation
Lung cancer [69]	Lung stagnation phlegm stasis syndrome, spleen deficiency phlegm dampness syndrome, yin deficiency phlegm heat syndrome, and qi-yin deficiency syndrome

Pancreatic cancer [70]	Blood stasis syndrome, spleen blood stasis syndrome, stomach qi up syndrome, and spleen yin deficiency syndrome

Liver cancer [71]	Qi stagnation and blood stasis syndrome, damp-heat accumulation syndrome, liver depression and spleen deficiency syndrome, and liver and kidney yin deficiency syndrome

Colorectal cancer [72]	Accumulated damp-heat syndrome, deficiency of both qi and blood syndrome, deficiency of liver and kidney yin syndrome, deficiency of spleen and kidney yang syndrome, and qi stagnation due to spleen deficiency syndrome

Gastric cancer [73]	Liver and stomach disharmony syndrome, qi stagnation and blood stasis syndrome, yin deficiency and internal heat syndrome, spleen and kidney yang deficiency syndrome, and qi and blood deficiency syndrome

Breast cancer [74]	Phlegm and blood stasis mutual syndrome, liver stagnation and qi stagnation syndrome, and Chong-Ren imbalance syndrome

Cervical cancer [75]	Deficiency of spleen and kidney yang syndrome, deficiency of liver and kidney yin syndrome, stagnation of liver and qi syndrome, and accumulation of heat toxin syndrome

Esophageal cancer [31]	Spittoon and qi blocking syndrome, phlegm and blood stasis syndrome, and qi deficiency and yang microsyndrome

## Data Availability

Data are openly available in a public repository.
